# Effects of Ringer’s sodium pyruvate solution on serum tumor necrosis factor-α and interleukin-6 upon septic shock

**DOI:** 10.12669/pjms.313.7170

**Published:** 2015

**Authors:** Wei Dong, Guannan Zhang, Feng Qu

**Affiliations:** 1 Wei Dong, Department of Critical Care Medicine, Second District, Shandong Jining No. 1 People’s Hospital, Jining 272011, China; 2 Guannan Zhang Shandong Jining No. 1 People’s Hospital, Jining 272011, China; 3 Feng Qu, Chief Physician, Department of Critical Care Medicine, Second District, Shandong Jining No. 1 People’s Hospital, Jining 272011, China

**Keywords:** Ringer’s sodium pyruvate solution, Septic shock, Tumor necrosis factor-α, interleukin-6

## Abstract

**Objective:**

To study the effects of Ringer’s sodium pyruvate solution on tumor necrosis factor-α (TNF-α) and interleukin-6 (IL-6) upon septic shock.

**Methods:**

Ninety emergency patients with septic shock were divided into a treatment group and a control group by random draw. The control group was resuscitated with 50 ml of compound sodium chloride (Ringer’s solution), and the treatment group was given 50 ml of Ringer’s sodium pyruvate solution. Both groups were basically treated.

**Results:**

All patients were successfully resuscitated. After treatment, extravascular lung water index, intrathoracic blood volume index, systemic vascular resistance index and cardiac index of the two groups were significantly improved compared with those before treatment (P<0.05). However, there were no significant inter-group differences at different time points (P>0.05). Blood lactic acid level, central venous oxygen saturation index and urine output were also improved after treatment, with significant inter-group differences (P<0.05). Serum TNF-α and IL-6 levels of both groups significantly decreased after treatment (P<0.05), and the levels of the treatment group were significantly lower than those of the control group (P<0.05). During 28 days of follow-up, the mortality rate of the treatment group (4.4%) was significantly lower than that of the control group (20.0%) (P<0.05).

**Conclusion:**

Patients with septic shock are complicated with disordered expressions of inflammatory factors. During resuscitation, Ringer’s sodium pyruvate solution can effectively promote blood circulation, mitigate inflammation and maintain acid-base equilibrium, thus decreasing the prognostic mortality rate.

## INTRODUCTION

Septic shock, which refers to a medical condition induced by severe infection and sepsis, is mainly responsible for the deaths in intensive care unit (ICU) and thus troubling doctors worldwide.^1^ When not treated timely, septic shock leads to cellular metabolism disorder, organ dysfunction, and even sudden death. Despite top-notch antibiotics, mechanical ventilation, monitoring and nutritional support, patients with septic shock are still prone to death.^2^,^3^ Besides, rational intervention and diagnosis are in need to dynamically observe the pathological and biological processes.^4^,^5^ Currently, septic shock is mainly treated by controlling infection, as well as by supplementing circulating blood volume, recovering tissue perfusion and improving cellular metabolism with fluid resuscitation.^6^,^7^

Intravenous fluid resuscitation can rapidly recover blood volume, blood pressure, cardiac function and urine output, which is now mainly performed by using Ringer’s solution to prevent adverse reactions.^8^ Inflammatory factors play important roles in septic shock-induced organ dysfunction.^9^ Once septic shock occurs, bacterial endotoxins and exotoxins as well as metabolites stimulate the release of proinflammatory cytokines such as tumor necrosis factor-α (TNF-α), interleukin-6 (IL-6) and oxygen radicals, resulting in toxic shock, organ dysfunction and death. As the key intermediate of glycolysis, pyruvic acid is the main constituent of energy metabolism and circulation and the center for metabolisms of carbohydrates, proteins and lipids in all tissues and organs of human body.^10^

Septic shock occurs based on uncontrollable inflammatory response induced by inflammatory mediators in early and advanced stages, during which considerable release of cytokines plays a crucial role. Cytokines have both pro- and anti-inflammatory effects which, if disturbed, will activate cascade reaction. Advanced-stage cytokines have long duration and interact with early-stage ones by positive feedback, being closely associated with the morality of septic shock.^11^ TNF-α, as an initiator of inflammation, induces the secretion of other cytokines such as IL-1, IL-6, IL-8 and CSF and cooperates with them in inflammatory response.^12^,^13^

On the other hand, sodium pyruvate dialysate can facilitate the glycometabolism of shock cells, enhance systemic alkalization and antioxidant capacity, and protect organs from lactic acidosis.^14^ Ringer’s sodium pyruvate solution, which replaces sodium lactate with 28 mM sodium pyruvate, combines their advantages and have cytoprotective effects.^15^ In this study, the effects of Ringer’s sodium pyruvate solution on serum TNF-α and IL-6 upon septic shock were evaluated.

## METHODS

### Subjects

Ninety patients with septic shock enrolled in ICU of our hospital from February 2008 to November 2013 were selected in this study. This study has been approved by the ethic committee of our hospital, and written consent was obtained from all patients. Diagnostic criteria for septic shock: Severely infected patients who had uncorrected, persistent low blood pressure levels (systolic pressure < 90 mmHg or decrease by 40 mmHg compared with normal level, MAP < 60-40 mmHg, capillary refill time > 2 s, cold limbs or mottled skin, low urine output) after sufficient fluid resuscitation, commonly accompanied by hypoperfusion or organ dysfunction.

### Inclusion criteria

In accordance with the diagnostic criteria for septic shock; 20-80 years old; with written consent.

### Exclusion criteria

ICU hospitalization stay length < 24 hour; use of drugs affecting immune function within six months; with autoimmune disease, acute cardiovascular disease, or HIV infection. The patients were divided into a treatment group and a control group by random draw (n=45), with similar gender, age, height, body weight and acute physiology and chronic health evaluation (APACHE) II score (P>0.05) (Table-I).

**Table-I:** Baseline clinical data.

Index	Treatment group (n=45)	Control group (n=45)	χ² or t	P
Gender (male/female)	25/20	24/21	0.067	>0.05
Age (years old)	56.33±4.12	56.29±5.01	0.045	>0.05
Body weight (kg)	60.39±10.38	60.57±9.32	0.293	>0.05
Height (cm)	165.39±11.67	165.02±12.00	0.193	>0.05
APACHE II score (point)	19.37±3.14	19.39±2.92	0.021	>0.05

### Resuscitation methods

All patients were treated according to their diseases and given sufficient anti-infective therapy and nutritional support. The control group was resuscitated by being intravenously injected with 50 ml of compound NaCl by using a microinjection pump for one hour (once every 12 h). By using the same method, the treatment group was resuscitated with 50 ml of Ringer’s sodium pyruvate solution (50 mM sodium pyruvate). PiCCO plus monitor (Pulsion, Germany) was employed to adjust the injection dose and speed. The patients should be supplemented with fluids timely when extravascular lung water index (EVLWI) < 14 ml/kg and intrathoracic blood volume index (ITVBI) < 1000 ml/m^2^. The fluid amount should be limited when EVLWI was lower than the normal level and ITVBI exceeded the normal level. When systolic pressure < 80 mmHg, additional vasoactive drugs were given. When EVLWI was higher than the normal level, urine-promoting therapy was given besides controlling fluid amount.

### Observation indices

Criteria for successful resuscitation: Cardiac index (CI) >4.5 L/(min·m^2^), oxygen index >600 ml/(min·m^2^), oxygen consumption index > 170 ml/(min·m^2^). Monitoring of hemodynamic indices: ITVBI, CI, systemic vascular resistance index (SVRI) and EVLWI were monitored before and two hour, 6 hour and 24 hour after treatment. Detection of central venous oxygen saturation, lactic acid level and urine output: Central venous oxygen saturation, lactic acid level and urine output were detected before and 24 hour after treatment.

Detection of TNF-α and IL-6 levels: Fasting peripheral blood (5 ml) was collected before and 24 h after treatment, left still and centrifuged at 2000 r/minutes for 20 minutes, from which the supernatant serum was collected and stored in a -80ºC refrigerator prior to use. Afterwards, the levels of TNF-α and IL-6 were detected with double-antibody sandwich enzyme-linked immunosorbent assay according to the instructions of kit (Beijing Jingmei Biotech Co., Ltd., China). Investigation on prognostic survival: All patients were followed up for 28 days to observe their survival.

### Statistical Analysis

All data were analyzed by SPSS 18.0. The means of categorical data were compared by t test and Wilcoxon rank-sum test. The numerical data were compared by Chi-square analysis. P<0.05 was considered statistically significant.

## RESULTS

### Hemodynamic indices

All patients were successfully resuscitated. ITVBI, SVRI and CI were improved two hour after treatment, with significant intra-group differences (P<0.05). EVLWI was also significantly improved six hour after treatment compared with that before treatment (P<0.05). However, there were no significant inter-group differences at different time points (P>0.05) (Table-II).

**Table-II:** Hemodynamic indices before and after treatment (n=45, x±s).

	Index	Before treatment	2 h after treatment	6 h after treatment	24 h after treatment
Treatment group	ITVBI (ml/m^2^)	729.25±80.85	834.85±127.32*	945.12±137.42*	932.45±131.89*
	CI (L/min•m^2^)	3.1±1.2	3.5±1.3*	3.4±1.1*	3.4±1.1*
	SVRI (dyn.s.cm-5m^2^)	856.3±110.9	893.3±132.5	1018.2±151.4*	1722.3±114.5*
	EVLWI (ml/kg)	6.3±0.9	7.8±2.6*	9.3±3.1*	8.7±2.9*
Control group	ITVBI (ml/m^2^)	730.38±81.34	874.95±116.91*	942.91±113.04*	933.93±100.34*
	CI (L/min•m^2^)	3.1±1.3	3.4±1.0*	3.3±1.3*	3.3±1.0*
	SVRI (dyn.s.cm-5m^2^)	856.3±893	912.1±172.1	1010.3±100.8*	1711.9±89.9*
	EVLWI (ml/kg)	6.3±0.9	7.7±2.5*	9.4±2.9	8.6±3.1

* Compared with the indices before treatment, P<0.05. ITVBI: intrathoracic blood volume index; CI: cardiac index; SVRI: systemic vascular resistance index; EVLWI: extravascular lung water index.

### Central venous oxygen saturation, lactic acid level and urine output

Blood lactic acid level, central venous oxygen saturation index and urine output were also improved after treatment, with significant inter-group differences (P<0.05) (Table-III).

**Table-III:** Central venous oxygen saturation, lactic acid level and urine output before and after treatment (n=45, x±s).

Group		Central venous oxygen saturation	Lactic acid level (mmol/L)	Urine output (ml/kg•h)
Treatment group	Before resuscitation	45.7±2.3	7.4±2.8	0.27±0.06Δ
	24 h after resuscitation	70.3±3.4*ΔΔ	3.1±1.6*Δ	0.51±0.10*ΔΔ
Control group	Before resuscitation	46.5±1.9	7.3±2.6	0.28±0.05Δ
	24 h after resuscitation	60.5±3.6*	4.1±1.2*	0.37±0.13*

* Compared with the values before treatment,

P<0.05;

Δ comparison between two groups after treatment, P<0.05.

### TNF-α and IL-6 levels

Serum TNF-α and IL-6 levels of both groups significantly decreased after treatment (P<0.05), and the levels of the treatment group were significantly lower than those of the control group (P<0.05) (Table-IV).

**Table-IV:** TNF-α and IL-6 levels before and after treatment (pg/ml, x±s).

Group	Case number (n)	TNF-α		IL-6	
		Before treatment	After treatment	Before treatment	After treatment
Treatment group	45	209.34±45.15	81.37±14.92	65.91±12.73	16.39±10.23
Control group	45	211.78±43.09	124.78±32.09	65.98±11.62	34.28±13.01
t		0.293	31.983	0.078	12.733
P		0.11	0.00	0.25	0.00

### Mortality rate

During 28 days of follow-up, the mortality rate of the treatment group (4.4%) was significantly lower than that of the control group (20.0%) (P<0.05) (Table-V).

**Table-V:** Morality rates 28 days after treatment.

Group	Case number (n)	Death	Morality rate
Treatment group	45	2	4.4%
Control group	45	9	20.0%
χ²			6.442
P			0.00

## DISCUSSION

Septic shock results in hypovolemic shock, plummet of blood flow rate and flow, decreased oxygen-carrying capacity of red blood cells, organ tissue hypoperfusion, and dramatic metabolic changes, especially glucose metabolic disorder and acid-base disequilibrium, thereby inducing cellular metabolic disorder and organ dysfunction, and even multiple organ failure upon progression.^16^ It is now well-established that septic shock pathologically results from ischemia, anoxia and reperfusion injury. Particularly, overproduction of active oxygen and nitroxides triggers systemic inflammatory response syndrome that renders septic shock from reversible to irreversible, being closely associated with prognosis.^17^,^18^

In the early stage of septic shock, performing anti-infection therapy in addition to fluid resuscitation can block or reduce the production and release of inflammatory mediators, which is of great significance to the inhibition of disease progression. Moreover, rational intervention and diagnosis are required to dynamically observe the pathological and biological processes.^19^ At present, septic shock is mainly treated by controlling infection, as well as by supplementing circulating blood volume, recovering tissue perfusion and benefiting cellular metabolism with fluid resuscitation.^20^ An ideal fluid for resuscitation should be able to rapidly control infection, to shorten the shock time, and to prevent all kinds of complications. Nevertheless, requiring a large volume, fluid resuscitation easily induces organ circulation-perfusion, coagulopathy, etc. Recently, Ringer’s solutions have been widely applied in experimental and clinical practice.^21^

Widely existing in human body, pyruvates are the intermediates of glycolysis and the metabolic centers of three essential nutrients. Animal studies have verified that sodium pyruvate can treat shock and protect vital organs (e.g. brain and bowels) from injury, particularly inhibiting the apoptosis of lung and brain cells and maintaining the intestinal mucosal barrier function. Exogenous supply of sodium pyruvate maintains tricarboxylic acid cycle by augmenting the activity of pyruvic acid, so considerable energy is released to stabilize hemodynamics.^22^ In this study, ITVBI, SVRI and CI were improved two hour after treatment, with significant intra-group differences (P<0.05). EVLWI was also significantly improved six hour after treatment compared with that before treatment (P<0.05). However, there were no significant inter-group differences at different time points (P>0.05). Hence, abnormal distribution of systemic blood flow upon septic shock led to absolute or relative lack of effective circulating blood volume. In other words, resuscitation with Ringer’s solution played a crucial role in treating septic shock and alleviating tissue perfusion. Treating patients with septic shock by Ringer’s solution resuscitation as early as possible can significantly improve ITVBI and EVLWI as well as correct CI and SI. Regardless, EVLWI and CVP, especially those of severe patients, are bound to increase, but the temporary lung water increase hardly affects oxygenation and respiratory function.

Pathologically speaking, septic shock is a complicated process manifested as hypotension that leads to severe prognosis by inducing insufficient oxygen supply and energy metabolism disorders in organs, tissues and cells.^7^ During metabolism and circulation, sodium pyruvate, through competitive inhibition, promotes the metabolism of the pentose phosphate pathway to generate NADPH and the recovery of glycometabolic oxidation. As a result, glycometabolic disorder is alleviated. Sodium pyruvate is superior to sodium lactate in correcting acidic environment at the early stage of severe shock because renal glycogen regeneration is subjected to compensatory enhancement Furthermore, sodium pyruvate prevents the generation of oxygen radicals by hindering the formation of peroxides, and eliminates them by reacting with H_2_O_2_ to yield CO_2_ and H_2_O.^23^ In this study, blood lactic acid level, central venous oxygen saturation index and urine output were also improved after treatment, with significant inter-group differences also (P<0.05), suggesting that Ringer’s sodium pyruvate solution evidently relieved acidosis and benefited the reversal of refractory shock.

Resuscitation of septic shock is necessarily accompanied by tissue, organ ischemic reperfusion injuries during which acute liver, cardiac and gastrointestinal injuries are directly and/or indirectly induced, activating the inflammatory cascade also. In healthy human and locally inflammatory patients, inflammatory mediators released by activated inflammatory cells exert defensive effects at the sites of inflammation. These mediators damage vascular endothelial cells, dilate small blood vessels, raise the vascular wall permeability and contracts blood vessels and smooth muscles of other parts. Accordingly, patients may die of severe septic shock typified by hypotension and multiple organ dysfunction. IL-10, IL-4 receptor antagonists and other soluble anti-inflammatory molecules are the main anti-inflammatory mediators, while TNF-α and IL-6 are potent proinflammatory factors. Terrible outcomes are inevitable once the inflammation balance is destroyed. If the proinflammatory effect surpasses the anti-inflammatory effect, inflammatory mediators intend to continuously proliferate and to cause damages. In the opposite case, the possible compensatory anti-inflammatory response syndrome results in immunoparalysis instead.^24^ Serum TNF-α and IL-6 levels of both groups herein significantly decreased after treatment (P<0.05), and the levels of the treatment group were significantly lower than those of the control group (P<0.05), indicating that Ringer’s sodium pyruvate solution inhibited the inflammatory response after septic shock, mitigated oxygen free radical-induced proinflammatory response, and enhanced free radical-scavenging capacity.

TNF-α functions in septic shock by elevating body temperature as an endogenous pyrogen; by inducing vasodilation as well as decreases in blood pressure and tissue perfusion through producing copious NO; by destructing the integrity of vascular barrier both NO-dependently and NO-independently, which increases capillary permeability, enhances plasma extravasation and reduces venous return; by inhibiting the fibrinolytic system, which promotes the hemorrhagic necrosis of vital organs and even disseminated intravascular coagulation during septic shock. IL-6 is produced by monocytes and macrophages in the presence of IL-1 during inflammatory response, and it also facilitates the proliferation of T cells in cooperation with TNF-α. Upon severe infections and traumas, the produced catecholamine can significantly increase the plasma level of IL-6.^25^

It has previously been reported that after shock is resuscitated by intravenous injection, blood pressure and urine output are recovered, whereas systemic inflammatory response is gradually aggravated.^4^ In this study, during 28 days of follow-up, the mortality rate of the treatment group (4.4%) was significantly lower than that of the control group (20.0%) (P<0.05), revealing that Ringer’s sodium pyruvate solution managed to improve the prognosis, probably because resuscitation promoted systemic blood circulation, recovered intestinal barrier function and decreased inflammatory factors. In the meantime, this solution successfully facilitated intestinal microcirculation, corrected acidosis and protected the function of intestinal mucosal barrier.

In summary, patients with septic shock are complicated with disordered expressions of inflammatory factors. During resuscitation, Ringer’s sodium pyruvate solution is capable of effectively promoting blood circulation, relieving inflammation and maintaining acid-base equilibrium, thereby lowering the prognostic mortality rate.

## References

[1] Chang HW, Kim KH, Hwang HY, Kim JS (2014). Role of mitral valve repair in infective endocarditis. J Heart Valve Dis.

[2] Pupelis G, Drozdova N, Mukans M, Malbrain ML (2014). Serum procalcitonin is a sensitive marker for septic shock and mortality in secondary peritonitis. Anaesthesiol Intensive Ther.

[3] Kalam K, Qamar F, Kumar S, Ali S, Baqi S (2014). Risk factors for carbapenem resistant bacteraemia and mortality due to gram negative bacteraemia in a developing country. J Pak Med Assoc.

[4] Meng X, Li J, Bai X, Hu S, Sheng Z (2014). [The effects of sodium pyruvate Ringer solution on hemodynamic and organ functions during shock stage in dogs with a 50% total body surface area full-thickness burn]. Zhonghua Wei Zhong Bing Ji Jiu Yi Xue.

[5] Dios S, Balseiro P, Costa MM, Romero A, Boltaña S, Roher N (2014). The Involvement of Cholesterol in Sepsis and Tolerance to Lipopolysaccharide Highlighted by the Transcriptome Analysis of Zebrafish (Danio rerio). Zebrafish.

[6] Matone J, Moretti AI, Apodaca-Torrez FR, Goldenberg A (2013). Ethyl-pyruvate reduces lung injury matrix metalloproteinases and cytokines and improves survival in experimental model of severe acute pancreatitis. Acta Cir Bras.

[7] Hamlin SK, Parmley CL, Hanneman SK (2014). Microcirculatory alterations in shock states. Crit Care Nurs Clin North Am.

[8] Dong Z, Jianxin Z, Haraguchi G, Arai H, Mitaka C (2014). Procalcitonin for the differential diagnosis of infectious and non-infectious systemic inflammatory response syndrome after cardiac operation. Zhonghua Wei Zhong Bing Ji Jiu Yi Xue.

[9] Gosmini R, Nguyen VL, Toum J, Simon C, Brusq JM, Krysa G (2014). The Discovery of I-BET726 (GSK1324726A), a Potent Tetrahydroquinoline ApoA1 Up-Regulator and Selective BET Bromodomain Inhibitor. J Med Chem.

[10] Ren H, Jiang J, Chu Y, Ding M, Qie G, Zeng J (2014). Study of the effects of high volume hemofiltration on extra vascular lung water and alveolar-arterial oxygen exchange in patients with septic shock. Zhonghua Wei Zhong Bing Ji Jiu Yi Xue.

[11] Gu X, Jin FG, Fu EQ, Li XY, Liu JL, Sun YN (2007). Effect of Cytokines in Pathogenesis of Acute Respiratory Distress Syndrome. Progress in Modern Biomedicine.

[12] Nishigaki F, Miyayasu K, Tsujimoto S, Manda T, Shimomura K (1994). Potentiation of the toxicity of tumor necrosis factor by tumors in mice. Circ Shock.

[13] Cain BS, Meldrum DR, Dinarello CA, Meng X, Joo KS, Banerjee A (1999). Tumor necrosis factor - alpha and interleukin - 1beta synergistically depress human myocardial function. Crit Care Med.

[14] Wang J, Guo X, Cao J, Zhang X, Zhang J, Sun D (2014). Prolonged pretreatment of mice with cholera toxin, but not isoproterenol, alleviates acute lethal systemic inflammatory response. Int Immunopharmacol.

[15] Sharma N, Venado A, Morrison J (2014). Protocol-based Treatment of Septic Shock, Fibrinolysis for Submassive Pulmonary Embolism, and Use of Corticosteroids in Acute Exacerbations of Chronic Obstructive Pulmonary Disease Requiring Mechanical Ventilation. Am J Respir Crit Care Med.

[16] Wang Z, Su F, Rogiers P, Vincent JL (2007). Beneficial effects of recombinant human activated protein C in a ewe model of septic shock. Crit Care Med.

[17] Rao XP, Zhu LQ, Lian HH (2006). Protective effects of glutamine on the intestinal mucosal barrier in young rabbits under hemorrhagic shock. Zhongguo Dang Dai Er Ke Za Zhi.

[18] do Nascimento P, Vaid SU, Hoskins SL, Espana JM, Kinsky MP, Kramer GC (2007). Hypertonic 15% sodium pyruvate offers no initial resuscitation advantage compared with 8% hypertonic NACl in sheep with multiple hemorrhages. Shock.

[19] Bai X, Yu W, Ji W, Lin Z, Tan S, Duan K (2014). Early versus delayed administration of norepinephrine in patients with septic shock. Crit Care.

[20] Chen H, Alam HB, Querol RI, Rhee P, Li Y, Koustova E (2006). Identification of expression patterns associated with hemorrhage and resuscitation: integrated approach to data analysis. J Trauma.

[21] Lee CJ, Lee RP, Subeq YM, Lee CC, Peng TC, Hsu BG (2009). Propofol protects against hemorrhagic shock-induced organ damage in conscious spontaneously hypertensive rats. Biol Res Nurs.

[22] Raffray L, Receveur MC, Beguet M, Lauroua P, Pistone T, Malvy D (2014). Severe delayed autoimmune haemolytic anaemia following artesunate administration in severe malaria: a case report. Malar J.

[23] Sriratanaviriyakul N, Nguyen LP, Henderson MC, Albertson TE (2014). Drug reaction with eosinophilia and systemic symptoms syndrome (DRESS) syndrome associated with azithromycin presenting like septic shock: a case report. J Med Case Rep.

[24] Lv J, Zhao HY, Liu F, An YZ (2012). The influence of lactate Ringer solution versus hydroxyethyl starch on coagulation and fibrinolytic system in patients with septic shock. Zhongguo Wei Zhong Bing Ji Jiu Yi Xue.

[25] Fioretto JR, Martin JG, Kurokawa CS, Carpi MF, Bonatto RC, Ricchetti SM (2008). Interleukin - 6 and pro- calcitonin in children with sepsis and septic shock. Cytokine.

